The article "Study on the Clinical Implications of NLR and PLR for Diagnosing Frailty in Maintenance Hemodialysis Patients and Their Correlations with Patient Prognosis" was published in 2022. Journal: J Healthc Eng.

# Study on the Clinical Implications of NLR and PLR for Diagnosing Frailty in Maintenance Hemodialysis Patients and Their Correlations with Patient Prognosis

**DOI:** 10.1155/2022/1267200

**Published:** 2022-01-12

**Authors:** Jun Wang, Lijuan Huang, Meichang Xu, Lei Yang, Xu Deng, Bei Li

**Affiliations:** ^1^Department of Nephrology, Nanjing Integrated Traditional Chinese and Western Medicine Hospital Affiliated with Nanjing University of Chinese Medicine, Nanjing 210014, Jiangsu Province, China; ^2^Department of Nephrology, Nanjing Hospital of Chinese Medicine Affiliated to Nanjing University of Chinese Medicine, Nanjing 210012, Jiangsu Province, China

## Abstract

**Objective:**

To explore the clinical implications of neutrophil-to-lymphocyte ratio (NLR) and platelet-to-lymphocyte ratio (PLR) for diagnosing frailty in patients with maintenance hemodialysis (MHD) and their correlations with patient prognosis.

**Methods:**

A total of 185 patients with MHD admitted to the hemodialysis center of our hospital were selected, 72 of whom were diagnosed with frailty according to the Chinese version of Tilburg Frailty Indicator (TFI). The relevant data were collected, and the influencing factors of frailty in MHD patients were analyzed by one-way analysis of variance (ANOVA) and multivariate logistic regression. The value of NLR and PLR in diagnosing frailty in MHD patients was observed, and patients' all-cause mortality was compared during the 3-year follow-up. The influences of different levels of NLR and PLR on the survival of MHD patients were investigated.

**Results:**

Multivariate regression analysis identified that serum albumin, dialysis adequacy, NLR, and PLR are independent risk factors for frailty in MHD patients (*P* < 0.05). The area under the receiver operating characteristic (ROC) curve of NLR and PLR in diagnosing frailty in MHD patients was 0.859 and 0.799, respectively. Compared with the nonfrailty group, the 3-year mortality was higher, and the 3-year survival rate assessed by survival analysis was lower in the frailty group (*P* < 0.05). Patients with high NLR and PLR levels showed a lower 3-year survival rate.

**Conclusions:**

Dialysis adequacy, serum albumin, NLR, and PLR are independently associated with frailty in MHD patients. NLR and PLR are of a certain diagnostic value for frailty in MHD patients. MHD patients with frailty have an unfavorable prognosis, as of those with high NLR and PLR levels.

## 1. Introduction

Currently, maintenance hemodialysis (MHD) is the most important renal replacement therapy for patients with end-stage renal disease (ESRD) [1]. With the prolongation of the survival time of MHD patients, they are prone to complications such as phosphorus-calcium metabolism disorder, energy and protein consumption, and sarcopenia due to the combined action of various factors [2, 3], which predispose patients to increased risk of frailty. A foreign study has shown that 60.7% of MHD patients suffer from frailty [4], and reports at home and abroad in recent years show that the incidence of frailty in MHD patients is 14%–73% [5]. Frailty leads to increased incidence of fractures, falls, hospitalization, and mortality [6]. Microinflammation is prevalent in MHD patients. It is shown that inflammation is the key pathogenesis leading to frailty in patients [7]. As novel inflammatory factors, neutrophil-to-lymphocyte ratio (NLR) and platelet-to-lymphocyte ratio (PLR) play an important role in the occurrence and development of diseases including coronary heart disease, myocardial infarction, and neoplastic diseases [8, 9]. In view of the current gap in the diagnosis and prognosis prediction of NLR and PLR in frailty of MHD patients, this study investigates the clinical implications of NLR and PLR for diagnosing frailty in MHD patients and their correlations with patient prognosis.

The article "Study on the Clinical Implications of NLR and PLR for Diagnosing Frailty in Maintenance Hemodialysis Patients and Their Correlations with Patient Prognosis" was published in 2022. Journal: J Healthc Eng.

## 2. Materials and Methods

### 2.1. General Information

The clinical data of 185 MHD patients (age: 32–80, mean age: 55.6 ± 13.5) treated in the outpatient department of Nanjing Integrated Traditional Chinese and Western Medicine Hospital and Nanjing Hospital of Chinese Medicine Affiliated to Nanjing University of Chinese Medicine from July 2015 to October 2018 were collected for retrospective analysis. The Ethics Committee at the Nanjing Integrated Traditional Chinese and Western Medicine Hospital approved the study protocol without reserves (ethics approval number: 2021–03). Inclusion criteria were as follows: meeting the diagnostic criteria of ESRD [2], dialysis for more than 6 months, age ≥18, and regular MHD 3 times per week. Exclusion criteria were as follows: hemodialysis (HD) treatment for acute renal failure, irregular MHD treatment due to economic or family reasons, malignant tumor(s), use of hormone or immunosuppressant therapy in recent 3 months, and infection in the last month.

### 2.2. Methods

The Chinese version of the Tilburg Frailty Indicator (TFI) (Cronbach's *α* coefficient = 0.686) [10], with a total score of 15 points and a score ≥5 indicating frailty, was used to evaluate the presence of frailty in patients. According to the results of TFI, 72 cases were assigned to the frailty group and 113 to the nonfrailty group. In addition, relevant literature and reports on frailty in MHD patients were searched, and the influencing factors were summarized to make a questionnaire. What is more, we collected patients' general data, clinical data, blood routine, and blood biochemical data (routine blood routine and blood biochemical tests were performed in the hemodialysis room before hemodialysis every 3 months, and the latest reports prior to patients' participating in this study were collected for analysis) for analysis. PLR and NLR were calculated based on the blood routine indexes of the included patients. PLR represents the neutrophil/lymphocyte ratio, and NLR represents the platelet/lymphocyte ratio.

The article "Study on the Clinical Implications of NLR and PLR for Diagnosing Frailty in Maintenance Hemodialysis Patients and Their Correlations with Patient Prognosis" was published in 2022. Journal: J Healthc Eng.

### 2.3. Outcome Measures

1. The influencing factors of frailty in MHD patients were determined by one-way analysis of variance (ANOVA) and binary logistic regression
2. The diagnostic value of PLR and NLR for frailty in MHD patients was observed
3. The 3-year mortality was observed and compared
4. The effects of different levels of NLR and PLR on the survival of MHD patients were analyzed

### 2.4. Statistical Processing

SPSS22.0 statistical software (Easy Bio (Beijing) Technology Co., Ltd., China) was used to analyze data. The normally distributed continuous variables were described as mean ± standard deviation (‾*X* ± SD), and the differences were analyzed by the *t*-test of independent samples (denoted by t). Nonnormally distributed measurement data were recorded as the median (lower and upper quartiles), and intergroup comparisons were performed by Mann–Whitney *U*-tests. The count data were tested by the Pearson chi-square test and expressed as *χ*^2^. Variables that differed in univariate analysis were screened, and the influencing factors of frailty in MHD patients were analyzed by multivariate binary logistic regression. After plotting the receiver operating characteristic (ROC) curves, the area under the ROC curves (AUROC) was calculated, with the values of 0.5–0.7 indicating small diagnostic utility, 0.7–0.9 indicating medium diagnostic utility, and >0.9 indicating high diagnostic utility. Patient survival was analyzed by the Kaplan–Meier method with the use of the log-rank test, and the multivariate analysis was performed using the Cox model. *P* values < 0.05 indicated that the differences were statistically significant.

## 3. Results

### 3.1. Comparison of General Information and Clinical Data

Among the 185 patients included, 72 patients had frailty, accounting for 38.92%. Patients in the frailty group were elder with higher NLR and PLR, while lower dialysis adequacy, serum albumin (SA), grip strength (GS), walking speed (WS), and midarm muscle circumference (MAMC) than the nonfrailty group (*P* < 0.05). In addition, there were no significant differences in sex, dialysis duration, education years, type 2 diabetes mellitus, coronary artery disease, hemoglobin, predialysis blood urea nitrogen, predialysis serum creatinine, uric acid, triglyceride, total cholesterol, high-density lipoprotein, low-density lipoprotein, blood potassium, blood calcium, blood phosphorus, body mass index, and upper arm circumference between the two groups (*P* > 0.05) as given in Table 1.

The article "Study on the Clinical Implications of NLR and PLR for Diagnosing Frailty in Maintenance Hemodialysis Patients and Their Correlations with Patient Prognosis" was published in 2022. Journal: J Healthc Eng.

### 3.2. Influencing Factors Related to Frailty in MHD Patients by Logistic Regression Analysis

The occurrence of frailty was used as the dependent variable (1 = occurrence; 0 = nonoccurrence), and the indicators which differed in the univariate analysis were selected for multivariate binary logistic regression analysis. It was found that dialysis adequacy, SA, NLR, and PLR were all risk factors leading to frailty in MHD patients as given in Table 2.

### 3.3. Diagnostic Value of NLR and PLR for Frailty in MHD Patients

The AUROC of NLR for diagnosing frailty in MHD patients was 0.859. When the cutoff value of NLR was 2.98, its Youden index, specificity, and sensitivity were 0.666, 0.805, and 0.861, respectively. The AUROC of PLR for diagnosing frailty in MHD patients was 0.799, and when the cutoff of PLR was 118.98, its Youden index, specificity, and sensitivity were 0.642, 0.850, and 0.792, respectively, as shown in Figure 1.

### 3.4. Correlations of NLR and PLR with Prognosis of MHD Patients

With the NLR diagnostic cutoff value of 2.98 as the dividing line, the patients were further assigned to the NLR high-expression group (*n* = 84) and NLR low-expression group (*n* = 95). Survival analysis showed that the survival rate of the NLR high-expression group was lower than that of NLR low-expression, with a statistical difference (*χ*2 = 19.922, *P* < 0.001). Similarly, the patients were assigned to high (*n* = 76) and low (*n* = 103) PLR expression groups, with the PLR diagnostic threshold of 118.98 as the dividing line. Survival analysis showed a significantly lower survival rate in patients with high PLR expression compared with those with low PLR expression (*χ*2 = 4.617, *P*=0.032), as shown in Figure 2.

### 3.5. Comparison of 3-Year Mortality

Six (1 in the frailty group and 5 in the nonfrailty group) of the 185 patients were lost to follow-up due to hospital referrals or other factors. Thirteen cases out of the 71 patients with frailty died within the 3 years of follow-up, with an incidence of 18.31%. While 9 cases among the 108 cases in the nonfrailty group died within 3 years, with an incidence of 8.33% (*P* < 0.05). The survival analysis revealed that the 3-year survival rate of the frailty group was significantly lower than that of the nonfrailty group (*χ*2 = 3.932, *P*=0.047). Multivariate COX proportional risk model analysis identified that NLR was an independent risk factor affecting the prognosis of MHD patients, as given in Tables 3 and 4 and Figure 3.

The article "Study on the Clinical Implications of NLR and PLR for Diagnosing Frailty in Maintenance Hemodialysis Patients and Their Correlations with Patient Prognosis" was published in 2022. Journal: J Healthc Eng.

## 4. Discussion

Frailty is a condition in which the decrease of physiological reserve and the dysfunction of multiple systems lead to the decline of the body's ability to cope with external conditions. In addition to the increase of vulnerability of the body, it can lead to an increase in the incidence of adverse events, resulting in adverse prognosis of patients [11]. MHD patients have an increased incidence of frailty due to both the disease itself and the treatment [12]. A foreign study showed that the incidence of frailty in MHD patients can reach 33.2% [13]. In the present study, 72 of the 185 enrolled patients with MHD in Nanjing had frailty with an incidence rate of 38.92%, which was similar to the above results.

The influencing factors of frailty in MHD patients were discussed in this study. The incidence of frailty increases with age and can reach 21.5% among the elderly in China [14]. Dialysis adequacy refers to the removal of excess water and toxins from the patient's body through HD to reach a comfortable state [15]. In a domestic study involving 120 MHD patients, dialysis adequacy was tested, and it was found that MHD patients with more adequate dialysis (i.e., urea clearance index ≥1.2) had a lower probability of muscle content decline and were less prone to frailty [14]. In addition, malnutrition and sarcopenia are common complications in MHD patients. Evidence has shown that MHD patients with hypoproteinemia are more susceptible to frailty, and the SA level is negatively correlated with the degree of frailty [15]. Another study holds that sarcopenia is the core mechanism of frailty, and GS, WS, and MAMC are important indexes to diagnose and evaluate sarcopenia [16, 17]. At present, the clinical etiology of frailty is still unclear, but studies have shown that chronic inflammation is the key mechanism leading to frailty [18]. Both NLR and PLR are important indicators of systemic inflammation. It is shown that NLR can be used as an independent risk factor for predicting renal failure in patients with stage 4 chronic kidney disease [19]. Under the stimulation of inflammation, megakaryocytic hyperplasia can be induced to increase the count of platelets, which will interact with endothelial cells and leukocytes to produce inflammatory factors, resulting in a vicious cycle. The onset of many diseases is associated with the increase of platelets [20]. Another study showed a correlation between platelet count and inflammatory status in MHD patients. PLR is an indicator reflecting the stability of platelets in the human body [21]. This study showed that the microinflammation of MHD patients with frailty was more obvious, which was related to the high expression of inflammatory factors in the microinflammatory state that promoted the occurrence of the disease and induced frailty. Regression analysis identified that in addition to NLR and PLR, SA and dialysis adequacy were also independent risk factors for frailty in MHD patients.

The article "Study on the Clinical Implications of NLR and PLR for Diagnosing Frailty in Maintenance Hemodialysis Patients and Their Correlations with Patient Prognosis" was published in 2022. Journal: J Healthc Eng.

Microinflammation is a common condition in patients with MHD. In this study, the diagnostic value of NLR and PLR for frailty in MHD patients was further studied. The results of ROC analysis determined that both NLR and PLR were of certain diagnostic value for frailty in MHD patients. At present, no study has explored the clinical implications of NLR and PLR for diagnosing frailty in MHD patients. Previous studies have shown a strong connection between inflammation and the occurrence and development of diseases such as sarcopenia, malnutrition, type 2 diabetes, and coronary heart disease [22], which may be related to the occurrence of inflammation-induced diseases and the body's susceptibility to frailty in the comorbid state.

In MHD patients with frailty, the risk of fracture, fall, hospitalization, and death increases significantly, leading to a decline in patients' quality of life and adversely affecting their prognosis [23]. Due to the disease itself and the fact that hemodialysis cannot completely replace renal function, patients are prone to frailty in the long-term hemodialysis process, which can induce cardiovascular events and affect their outcomes [24]. This study also showed a higher 3-year mortality in MHD patients with frailty. NLR and PLN levels have been indicated to be of certain predictive value for the clinical progression and prognosis of patients with osteosarcoma [25]. In another study, NLR and PLN could predict the survival of patients with lower limb arteriosclerosis obliterans [26]. This study further investigated the influence of different levels of NLR and PLR on the prognosis of MHD patients. It was found that MHD patients with high NLR and PLR levels had decreased survival and unfavorable prognosis, which may be related to the persistence of chronic inflammatory state inducing other diseases to exert an influence on patient prognosis. Finally, COX multivariate analysis showed that NLR was an independent risk factor affecting the prognosis of MHD patients. Zhang et al. [27] pointed out in their study that a higher level of NLR rather than PLR could predict the risk of cardiovascular death in MHD patients by predicting erythropoietin responsiveness, which is similar to our results.

The article "Study on the Clinical Implications of NLR and PLR for Diagnosing Frailty in Maintenance Hemodialysis Patients and Their Correlations with Patient Prognosis" was published in 2022. Journal: J Healthc Eng.

With the extended life span of MHD patients, the incidence of experiencing frailty is also on the rise, which deserves more attention from the clinic. Clinical workers should pay attention to the monthly blood routine testing of MHD patients and evaluate whether the microinflammatory state in patients with elevated NLR and PLR is associated with frailty, so as to take intervention measures such as nutritional intake and dialysis adequacy as early as possible. Referring to the previous research, we began to carry out exercise combined with nutritional support intervention therapy for MHD patients with frailty, searched for exercises suitable for MHD patients such as resistance exercise and Baduanjin, and set up a special nutritional support group to evaluate the nutritional status of patients and give individualized diet intervention, all of which can reduce the microinflammatory factors in patients to a certain extent and correct the patients' frailty.

The novelty of this study lies in that it not only confirmed the diagnostic and prognostic value of NLR and PLR in MHD but also proved the correlations of the two with the occurrence of frailty and the prognosis of MHD patients from multiple perspectives, such as related factors of frailty, diagnostic value in frailty, patient prognosis, and related influencing factors, which provides new clinical markers for the diagnosis and prognosis prediction of MHD patients and provides a new clinical reference for the prevention of frailty and poor prognosis in MHD patients.

Shortcomings and prospects: the sample size of this study is small, which can be further expanded to observe the influence of NLR and PLR on the diagnosis and prognosis of MHD patients with frailty.

## 5. Conclusion

To sum up, dialysis adequacy, SA, NLR, and PLR are independently associated with frailty in MHD patients. NLR and PLR are of certain clinical implications for diagnosing frailty in MHD patients. MHD patients combined with frailty are accompanied by poor prognosis, as of those with high NLR and PLR levels.

## Figures and Tables

**Figure 1:** ROC curve of NLR and PLR in diagnosing frailty in MHD patients. NLR, neutrophil-to-lymphocyte ratio; PLR, platelet-to-lymphocyte ratio.

**Figure 2:** Correlation of NLR and PLR with prognosis of MHD patients. (a) Survival curves of patients with high and low NLR expression levels. (b) Survival curves of patients with high and low PLR expression levels. NLR, neutrophil-to-lymphocyte ratio; PLR, platelet-to-lymphocyte ratio.

**Figure 3:** Survival curves of two groups of patients within 3 years.

**Table 1:** Comparison of related influencing factors of frailty in patients with 1MHD.

Categories	Frailty group (*n* = 72)	Nonfrailty group (*n* = 113)	*χ* ^2^/*t*/*Z* value	*P*
Male (*n* (%))	31 (43.06)	57 (50.44)	0.962	0.327
Age (years)	59.4 ± 13.7	53.2 ± 13.9	3.261	0.001
Dialysis duration (months)	66.94 (35.12, 88.72)	67.22 (34.21, 86.23)	0.573	0.632
Education years	8.65 ± 2.67	8.94 ± 2.86	0.582	0.552
Dialysis adequacy	1.43 ± 0.26	1.66 ± 0.27	5.726	<0.001
Type 2 diabetes mellitus (*n* (%))	28 (38.89)	31 (27.43)	2.657	0.103
Coronary artery disease (*n* (%))	14 (19.44)	19 (16.81)	0.208	0.649
SA (g/L)	37.16 ± 4.01	40.41 ± 3.25	6.058	<0.001
Hemoglobin (g/L)	107.62 ± 19.81	112.14 ± 15.47	1.734	0.085
Predialysis blood urea nitrogen (mmol/L)	25.74 ± 7.25	26.78 ± 7.36	0.943	0.347
Predialysis serum creatinine (umol/L)	583.82 (252.34, 762.12)	629.72 (272.67, 782.45)	1.432	0.156
Uric acid (umol/L)	463.24 ± 74.59	446.87 ± 71.26	1.496	0.136
Triglyceride (mmol/L)	1.71 (1.17, 2.34)	1.84 (1.12, 2.19)	0.675	0.485
Total cholesterol (mmol/L)	3.84 ± 0.79	3.92 ± 0.73	0.451	0.704
High-density lipoprotein (mmol/L)	1.01 ± 0.33	1.09 ± 0.36	1.522	0.130
Low-density lipoprotein (mmol/L)	3.38 ± 0.74	3.42 ± 0.71	0.368	0.714
Blood potassium (mmol/L)	4.74 ± 0.78	4.52 ± 0.74	1.930	0.055
Blood calcium (mmol/L)	2.04 ± 0.21	2.07 ± 0.23	0.894	0.372
Blood phosphorus (mmol/L)	1.92 ± 0.48	1.85 ± 0.49	0.955	0.341
NLR	4.18 ± 1.02	2.55 ± 0.95	11.091	<0.001
PLR	129.96 ± 12.62	112.62 ± 13.36	8.787	<0.001
Body mass index (kg/m^2^)	20.26 ± 2.58	21.01 ± 2.76	1.823	0.07
GS (kg)	20.11(14.32, 21.21)	28.72 (19.21, 36.72)	4.785	<0.001
WS (m/s)	0.65 ± 0.26	0.76 ± 0.25	2.921	0.004
Bicep's circumference (mm)	28.62 ± 2.31	29.11 ± 3.24	1.115	0.126
MAMC (mm)	21.62 ± 2.74	23.08 ± 2.72	3.548	<0.001

SA, serum albumin; NLR, neutrophil-to-lymphocyte ratio; PLR, platelet-to-lymphocyte ratio; GS, grip strength; WS, walking speed; MAMC, midarm muscle circumference.

The article "Study on the Clinical Implications of NLR and PLR for Diagnosing Frailty in Maintenance Hemodialysis Patients and Their Correlations with Patient Prognosis" was published in 2022. Journal: J Healthc Eng.

**Table 2:** Logistic regression analysis of influential factors related to frailty in MHD patients.

Variables	*β*	SE	Wald value	OR value (95% CI)	*P*
Constants	13.623	6.903	3.894	—	0.048
Age (years)	0.004	0.042	0.007	1.004 (0.925–1.089)	0.933
Dialysis adequacy	−3.506	1.439	5.937	0.030 (0.002–0.504)	0.015
SA (g/L)	−0.658	0.178	13.693	0.518 (0.365–0.734)	<0.001
NLR	2.022	0.429	22.188	7.554 (3.257–17.523)	<0.001
PLR	0.131	0.033	16.252	1.140 (1.070–1.216)	<0.001
GS (kg)	−0.073	0.048	2.305	0.929 (0.846–1.022)	0.129
WS (m/s)	−1.527	1.281	1.42	0.217 (0.012–2.676)	0.233
MAMC (mm)	−0.184	0.142	1.674	0.832 (0.629–1.099)	0.196

SA, serum albumin; NLR, neutrophil-to-lymphocyte ratio; PLR, platelet-to-lymphocyte ratio; GS, grip strength; WS, walking speed; MAMC, midarm muscle circumference.

**Table 3:** Comparison of 3-year mortality.

Groups	Death within 1 year	Death within 2 years	Death within 3 years
Frailty group (*n* = 71)	4 (5.63)	8 (11.27)	13 (18.31)
Nonfrailty group (*n* = 108)	1 (0.93)	4 (3.70)	9 (8.33)
*χ* ^2^	3.491	3.919	3.955
*P*	0.061	0.048	0.047

**Table 4:** COX multivariate analysis of prognosis in MHD patients.

Variables	*β*	SE	Wald	HR value (95% CI)	*P*
NLR	0.972	0.248	15.419	2.644 (1.627–4.295)	<0.001

NLR, neutrophil-to-lymphocyte ratio.

## Data Availability

The labeled datasets used to support the findings of this study are available from the corresponding author upon request.

## References

[1] Kramer A., Pippias M., Stel V. S. (2016). Renal replacement therapy in europe: a summary of the 2013 era-edta registry annual report with a focus on diabetes mellitus. *Clinical Kidney Journal*.

[2] Lai S., Muscaritoli M., Andreozzi P. (2019). Sarcopenia and cardiovascular risk indices in patients with chronic kidney disease on conservative and replacement therapy. *Nutrition*.

[3] Sabatino A., Piotti G., Cosola C., Gandolfini I., Kooman J. P., Fiaccadori E. (2018). Dietary protein and nutritional supplements in conventional hemodialysis. *Seminars in Dialysis*.

[4] Yoneki K., Kitagawa J., Hoshi K. (2019). Association between frailty and bone loss in patients undergoing maintenance hemodialysis. *Journal of Bone and Mineral Metabolism*.

[5] Lee S. Y., Yang D. H., Hwang E. (2017). The prevalence, association, and clinical outcomes of frailty in maintenance dialysis patients. *Journal of Renal Nutrition*.

[6] Takeuchi H., Uchida H. A., Kakio Y. (2018). The prevalence of frailty and its associated factors in Japanese hemodialysis patients. *Aging and disease*.

[7] Fulop T., Witkowski J. M., Olivieri F., Larbi A. (2018). The integration of inflammaging in age-related diseases. *Seminars in Immunology*.

[8] Serban D., Papanas N., Dascalu A. M. (2021). Significance of neutrophil to lymphocyte ratio (nlr) and platelet lymphocyte ratio (plr) in diabetic foot ulcer and potential new therapeutic targets. *The International Journal of Lower Extremity Wounds*.

[9] de Jong M. C., Mihai R., Khan S. (2021). Neutrophil-to-lymphocyte ratio (nlr) and platelet-to-lymphocyte ratio (plr) as possible prognostic markers for patients undergoing resection of adrenocortical carcinoma. *World Journal of Surgery*.

[10] Nixon A. C., Bampouras T. M., Pendleton N., Woywodt A., Mitra S., Dhaygude A. (2018). Frailty and chronic kidney disease: current evidence and continuing uncertainties. *Clinical Kidney Journal*.

[11] Kluszczynska M., Mlynarska A. (2021). Influence of frailty syndrome on patient prognosis after coronary artery bypass grafting. *Advances in Clinical and Experimental Medicine*.

The article "Study on the Clinical Implications of NLR and PLR for Diagnosing Frailty in Maintenance Hemodialysis Patients and Their Correlations with Patient Prognosis" was published in 2022. Journal: J Healthc Eng.

[12] Sy J., McCulloch C. E., Johansen K. L. (2019). Depressive symptoms, frailty, and mortality among dialysis patients. *Hemodialysis International*.

[13] Hanson C. S., Chapman J. R., Craig J. C. (2017). Patient experiences of training and transition to home haemodialysis: a mixed-methods study. *Nephrology*.

[14] Lin Y. L., Liou H. H., Lai Y. H. (2018). Decreased serum fatty acid binding protein 4 concentrations are associated with sarcopenia in chronic hemodialysis patients. *Clinica Chimica Acta*.

[15] Bharati J., Jha V. (2020). Achieving dialysis adequacy: a global perspective. *Seminars in Dialysis*.

[16] Lu X., Zhang J., Wang S., Yu Q., Li H. (2020). High erythropoiesis resistance index is a significant predictor of cardiovascular and all-cause mortality in Chinese maintenance hemodialysis patients. *Mediators Inflamm*.

[17] Metsemakers W., Morgenstern M., McNally M. A. (2018). Fracture-related infection: a consensus on definition from an international expert group. *Injury*.

[18] Yao C., Narumiya S. (2019). Prostaglandin-cytokine crosstalk in chronic inflammation. *British Journal of Pharmacology*.

[19] Yuan Q., Wang J., Peng Z. (2019). Neutrophil-to-lymphocyte ratio and incident end-stage renal disease in Chinese patients with chronic kidney disease: results from the Chinese cohort study of chronic kidney disease (c-stride). *Journal of Translational Medicine*.

[20] Marcoux G., Laroche A., Espinoza Romero J., Boilard E. (2021). Role of platelets and megakaryocytes in adaptive immunity. *Platelets*.

[21] Kara A. V., Soylu Y. E. (2019). The relationship between vitamin d and inflammatory markers in maintenance hemodialysis patients. *International Urology and Nephrology*.

[22] Massiot N., Lareyre F., Voury-Pons A. (2019). High neutrophil to lymphocyte ratio and platelet to lymphocyte ratio are associated with symptomatic internal carotid artery stenosis. *Journal of Stroke and Cerebrovascular Diseases*.

[23] Iwata Y., Okushima H., Takatsuka T. (2020). Duration of predialysis nephrological care and mortality after dialysis initiation. *Clinical and Experimental Nephrology*.

[24] Saghir Afifeh A. M., Verdoia M., Nardin M. (2021). Determinants of vitamin d activation in patients with acute coronary syndromes and its correlation with inflammatory markers. *Nutrition, Metabolism, and Cardiovascular Diseases*.

[25] Xia W.-K., Liu Z.-L., Shen D., Lin Q.-F., Su J., Mao W.-D. (2016). Prognostic performance of pre-treatment nlr and plr in patients suffering from osteosarcoma. *World Journal of Surgical Oncology*.

[26] Ye M., Qian X., Guo X. (2020). Neutrophil-lymphocyte ratio and platelet-lymphocyte ratio predict severity and prognosis of lower limb arteriosclerosis obliterans. *Annals of Vascular Surgery*.

The article "Study on the Clinical Implications of NLR and PLR for Diagnosing Frailty in Maintenance Hemodialysis Patients and Their Correlations with Patient Prognosis" was published in 2022. Journal: J Healthc Eng.

[27] Zhang J., Lu X., Wang S., Li H. (2021). Neutrophil-to-lymphocyte ratio and erythropoietin resistance among maintenance hemodialysis patients. *Blood Purification*.

